# Using Healthcare Resources Wisely: A Predictive Support System Regarding the Severity of Patient Falls

**DOI:** 10.1155/2022/3100618

**Published:** 2022-08-01

**Authors:** Hsi-Hao Wang, Chun-Che Huang, Paul C. Talley, Kuang-Ming Kuo

**Affiliations:** ^1^Department of Healthcare Quality, E-Da Hospital, Kaohsiung 82445, Taiwan; ^2^Department of Healthcare Administration, I-Shou University, Kaohsiung 82445, Taiwan; ^3^Department of Applied English, I-Shou University, Kaohsiung 84001, Taiwan; ^4^Department of Business Management, National United University, Miaoli 360301, Taiwan

## Abstract

**Background:**

An injurious fall is one of the main indicators of care quality in healthcare facilities. Despite several fall screen tools being widely used to evaluate a patient's fall risk, they are frequently unable to reveal the severity level of patient falls. The purpose of this study is to build a practical system useful to predict the severity level of in-hospital falls. This practice is done in order to better allocate limited healthcare resources and to improve overall patient safety.

**Methods:**

Four hundred and forty-six patients who experienced fall events at a large Taiwanese hospital were referenced. Eight predictors were used to ascertain the severity of patient falls solely based on the above study population. Multinomial logistic regression, Naïve Bayes, random forest, support vector machine, eXtreme gradient boosting, deep learning, and ensemble learning were adopted to establish predictive models. Accuracy, F1 score, precision, and recall were utilized to assess the models' performance.

**Results:**

Compared to other learners, random forest exhibited satisfying predictive performance in terms of all metrics (accuracy: 0.844, F1 score: 0.850, precision: 0.839, and recall: 0.875 for the test dataset), and it was adopted as the base learner for a severity-level predictive system which is web-based. Furthermore, age, ability of independent activity, patient sources, use of assistive devices, and fall history within the past 12 months were deemed the top five important risk factors for evaluating fall severity.

**Conclusions:**

The application of machine learning techniques for predicting the severity level of patient falls may result in some benefits to monitor fall severity and to better allocate limited healthcare resources.

## 1. Introduction

Falls are the second leading cause of death by unintentional or accidental injuries worldwide [1]. An estimated 37.3 million falls critical enough to necessitate medical attention occur each year, and about 646,000 fatal falls occur annually [1]. An injurious fall is considered to be one of the main indicators of care quality in monitoring patient safety in healthcare facilities [2]. Ensuring patient safety in hospitals has remained a major public health concern [2–4]. Individuals who had fall events within healthcare environments regarding patient safety are of extreme importance to monitor and necessary to prevent accidental and injurious falls [5]. In addition, when a fall occurs, patients have different levels of injury, prolonging their treatment periods and increasing healthcare costs, perhaps even causing death [3, 6, 7].

Thus far, several tools such as the Morse Fall Scale [8], the St. Thomas Risk Assessment Tool in Falling Elderly Inpatients [9], and the Hendrich II Fall Risk Model [10] have been applied to evaluate fall risk. These tools have surely provided valuable assistance to existing fall measures by identifying all susceptible patients. Healthcare facilities then foster and engage in coping strategies to diminish the occurrence of these plausible fall events among their patient population. This approach may be feasible with sufficient healthcare resources. During particular occasions such as the COVID-19 pandemic, all healthcare resources are so limited that it is not possible to allocate abundant resources in detecting and handling all fall events as once before. Therefore, these fall risk screening tools will have been more valuable and comprehensive if they are able to predict the severity of fall events. By knowing the severity level, healthcare facilities can better allocate limited resources and use resources more wisely for the most needy patients [11].

Prior studies have done specific machine learning methods for selecting factors and classification modes according to incident reports and predicted the probability of adverse event occurrence in healthcare facilities [12–15]. However, there is a dearth of studies evaluating the severity level of patient falls, not to mention the inclusion of machine learning techniques. In order to better improve patient safety practices, a user-friendly prediction system for screening patients of plausible severe fall events is critically required. Therefore, the purpose of this study (*see*Figure 1) is to develop a useable predictive support system based on machine learning techniques, which can facilitate the assessment of the prior severity level of patient falls in healthcare facilities.

### 1.1. Related Works

To date, previous studies have identified various fall risk factors inherent to hospital environments. For example, Liu et al. [16] found several factors such as age, unassisted movement, impaired mobility, and fall history within the past 12 months as being imperative to the prediction of patient falls. They were however unable to identify whether having any companions present at the time of fall acts as a risk or mitigating factor. Cho et al. [17] contrasted three fall risk assessment scales (i.e., Morse Fall Scale, The John Hopkins Hospital fall risk assessment tool, and Hendrich II fall risk model) and indicated important risk factors such as fall history, ambulatory aid, gait, mental status, medication, requirement of assistance or supervision, symptomatic depression, altered elimination, and dizziness. In their study of fall risk factors of inpatients, Najafpour et al. [4] showed important risk factors such as longer length of stay, using chemotherapy drugs, anticonvulsants, sedatives, angiotensin-converting enzyme inhibitors, benzodiazepines, balance condition, visual acuity, and manual transfer aid. They were however unable to prove fall history being a significant risk factor in patient care. Ozturk et al. [18] found fall-related factors for emergency patients including being physically active before the fall event, being between 65 and 79 years of age, having chronic diseases, and being on benzodiazepine and other specific medications. Aryee et al. [19] confirmed that recent surgery was protective, joint replacement, psychotropic agents, male gender, and history of fall were critical fall risk factors for surgical patients. Another study reported that rates of fall injury diagnoses in the emergency department were generally higher among older women [20]. Chen et al. [21] demonstrated independent risk factors for falls among aged inpatients including insomnia at the time of admission, new episodes of leg weakness, postural hypotension, newly prescribed hypnotics during admissions, more than one fall event history within the previous year, and caregiver's accompaniment. These studies have paved the foundation on this important topic. In accordance with prior evidence, we can see these identified fall risk factors being quite diversified in nature and no consensus on this issue has yet to be reached. Furthermore, the studies mentioned adopted a traditional statistical model requiring strict assumptions for analyzing the data [22].

Thus far, several studies have used machine learning to approach issues related to patient safety (*see*Table 1). For example, Ong et al. [23] adopted Naïve Bayes and support vector machine to develop text classifiers for automatically detecting extreme-risk adverse events taken from clinical incident reports. Their results showed that support vector machine performed best with F-measure = 0.86, precision = 0.88, recall = 0.83, and area under the receiver operating characteristic curve (AUC) = 0.92 in identifying incident types. Cheng and Zhao [25] proposed a heterogeneous, network-assisted inference framework to support for forecasting drug-drug interactions. They applied five algorithms including decision tree, Naïve Bayes, k-nearest neighbor, support vector machine, and logistic regression to establish the proposed framework. Support vector machine demonstrated the best performance with an AUC of 0.67. In order to screen hazardous cases related to electronic health records, Marella et al. [12] tested several algorithms comprising Naïve Bayes kernel, Naïve Bayes, k-nearest neighbor, and rule reduction. They found that Naïve Bayes kernel performed best in terms of AUC (0.84) and accuracy (0.75).

These prior efforts surely add knowledge and improve our understanding of patient safety. A literature review, however, demonstrates research gaps regarding applied machine learning techniques and patient safety issues. First, these prior studies have not yet investigated the severity level of patient falls. Second, most studies focus on assessing the types of patient safety incidents [12, 13, 15, 16, 23, 26, 29]. The characteristics of various patient safety incidents remain diversified, and it is therefore difficult to reach a satisfying solution. Instead, studies may wish to further identify a specific incident such as patient fall event in order to gain a better understanding on the nature of such an incident. Third, evidence shows that support vector machine is frequently adopted as algorithm for establishing predictive models; however, this allows room for testing how other algorithms might perform with regard to patient safety problems.

## 2. Material and Methods

### 2.1. Study Population and Setting

Data were obtained from the Taiwan Patient-safety Reporting System (TPRS) [30] of a large hospital in southern Taiwan from 2019 to 2020. TPRS is an incident report system that can collect patient adverse events including medication, falls, operations, blood transfusions, health care, and public accidents. Our study focused on fall adverse events because the collected data are more comprehensive than the other types of adverse events. Eligibility criteria were that a patient must (1) be aged over 20 and (2) belongs to a fall event. The Institutional Review Board of E-Da hospital permitted the study protocol and waived informed consent (EMRP-109-159).

### 2.2. Measures

Patients' baseline information comprising gender, age, patient sources, fall history within the past 12 months, ability to perform an independent activity (assessed by means of the Barthel index), companionship (such as family members, relatives, friends, or caregivers being present at the event), and use of assistive devices (defined as a device that assists patients in accompanying day-to-day functions [21]) were collected and used as features for building the predictive model. The relative severity of patient falls is the target of the predictive model.  Table 2 shows the operational definitions of variables included in this study.

### 2.3. Experimental Setup

In order to build a machine learning model to forecast the severity of fall adverse events, we adopted R 4.1.2 [31] for data analysis and Python 3.7 [32] with scikit-learn 1.1.0 [33] for building predictive models. We chose seven learners including multinomial logistic regression, Naïve Bayes, random forest, support vector machine, eXtreme gradient boosting, deep learning, and ensemble learning to construct the predictive model. These learners were chosen for comparative purpose, and these learners are frequently used in building healthcare predictive models with good performance [34]; Chen et al. [35–37]. Regarding ensemble learning, we adopted the stacking approach because two other ensemble approaches, including bagging and boosting, were implemented by random forest and eXtreme gradient boosting. We used logistic regression as the meta-model. Models based on multinomial logistic regression, Naïve Bayes, random forest, support vector machine, eXtreme gradient boosting, and deep learning with better performance were then chosen as the base models since the rationale for using the stack approach is to learn how best to combine the predictions from multiple well-performed machine learning algorithms [38].

We adopted a random search approach to automatically determine the optimal combinations of parameters for the selected machine learning algorithms in order to reach a better prediction performance (*see*Table 3). We used the 2019 data as a training dataset and the 2020 data as the test dataset, aiming to improve the model's accuracy and to diminish any possible overfitting issues [22]. Since the collected data were imbalanced in the target variable, a synthetic minority over-sampling technique, for the training dataset, was leveraged by under-sampling the adequate class and over-sampling the inadequate class in order to improve the model performance [39]. Further, we applied a 10-fold cross-validation method to assess the six learners with the training dataset in order to better estimate the model performance. Mean and standard deviation of performance metrics are calculated.

### 2.4. Performance Measure

Since the target in this study is three class, more suitable metrics including accuracy, F1-score, precision, and recall are adopted to assess the performance of predictive models [40]. These four metrics are based on a confusion matrix which includes four predicted results: true positive, false positive, false negative, and true negative; as such, the four metrics can then be derived [22]. When interpreting the model performance, the closer to the value of 1 is considered the better for all metrics concerned [22].

## 3. Results

### 3.1. Data Profiles

A total of 446 patients who experienced falls were included, 209 patients in 2019 and 237 in 2020. The distributions of patient's demographics are similar in 2019 and 2020. Among these cases, males were more represented than females (*see*Table 4). Most patients were aged 51–80 years, while most subjects belonged to inpatient care. In addition, 73.21% and 74.26% of patients had fallen in the past 12 months in 2019 and 2020, respectively; over 90% of patients were labeled at high risk of falling. Approximately 61.24% and 59.49% of patients belonged to the group who were partially dependent on their family members or friends in the prior two years to the event, and 75.6% and 72.15% of them did not have usual companions present. Further, in both years, 46.89% and 45.57% of the patients used assistive devices. Regarding the severity of fall events, 47.85% and 54.01% of patients had severe adverse effects, 15∼16% of patients had mild adverse effects, and more than 30% of patients had no adverse effects whatsoever.

### 3.2. Model Performance

Table 5 shows the performance results of seven learners including multinomial logistic regression (MLR), Naïve Bayes (NB), random forest (RF), support vector machine (SVM), eXtreme gradient boosting (XGBoost), deep learning (DL), and Stacking for the training and test dataset, respectively. Accuracy, F1-score, precision, and recall were used to assess the performance of those learners. Based on the results of 10-fold cross-validation, RF, SVM, XGBoost, and DL were included in the Stacking as the base models while MLR and NB were not included due to all four metrics being lower than 0.5 for both learners (*see*Table 5).

As demonstrated in Table 5, RF has the best accuracy score (0.783), followed by XGBoost (0.778), SVM (0.771), Stacking (0.756), and DL (0.721). In terms of F1-score, RF has the highest score (0.784), followed by XGBoost (0.779), SVM (0.771), Stacking (0.754), and DL (0.720). As for precision, RF has the highest score (0.785), followed by XGBoost (0.781), SVM (0.774), Stacking (0.760), and DL (0.735). Regarding recall score, RF still has the highest score (0.788), followed by XGBoost (0.784), SVM (0.776), Stacking (0.763), and DL (0.725). In sum, RF performs better than the remaining learners for the training dataset. We further validated our built models with a test dataset. RF still outperforms the other learners in terms of all four metrics.

A comprehensive assessment of the performance for the selected learners based on four metrics shows that RF performs better than MLR, NB, SVM, XGBoost, DL, and Stacking. The area under the receiver operating characteristic curve and confusion matrix of the RF learner for the test dataset are illustrated in Figures 2 and 3, respectively. Further, there is no clear evidence of overfitting based on the performance metrics of training and test datasets in addition to MLR and NB [22].

### 3.3. Comparison with Benchmark Models

To better support our findings, we compared the results of the performance of our built predictive model based on random forest learner with the results of the Morse Fall Scale [8]. The target variable in this study is three class indicating the severity of fall events (no, mild, and severe adverse effect) which is inconsistent with the three risk levels (no, low, and high risk) of the Morse Fall Scale. Moreover, severe adverse events and high Morse fall risk scores were less frequently observed in patients who experienced falls. We therefore segment the severity of fall events into two classes, namely no adverse effect and possible adverse effect (including mild and severe adverse effect), and segment the Morse risk levels into two levels, namely no risk and possible risk (including low and high risk). An accuracy score of about 0.57, better than randomly guessing, was obtained by comparing the predicted results of the test dataset with the re-coded Morse fall risk levels. This result is expected because the primary purpose of our study is to predict the severity of fall events rather than the fall risk. Further, high risk of falling does not mean severe adverse effect when patients do happen to fall.

### 3.4. Feature Importance and Model Explainability

Apart from comparing the performance of learners, we also graded the feature importance based on Shapley additive explanations (SHAP) values [41]. Higher SHAP value indicates more strength of features' contribution to the prediction results [41]. As shown in Figure 4, the top five important features for predicting severe adverse effect included age, ability of independent activity, use of assistive devices, fall history within the past 12 months, and patient source.

We further analyzed the relationship between features and predicted adverse effect based on the beeswarm plot. As shown in Figure 5, we can acquire some insights such as higher age, higher dependence, use of assistive devices, and patients without fall history within the past 12 months all lead to higher probability of severe adverse effect.

### 3.5. Severity-of-Fall Prediction System

Based on the performance of seven learners, we chose RF as the primary learner for developing a severity-of-fall prediction system, which can be considered as a supporting system adding to patient safety. To ensure this support system can be deployed in differing computer platforms, we adopted a representational state transfer (RESTful) application programming interface based on a Flask package [42] to establish application efficacy. Based on the RESTful approach, users can use the prediction support system from browsers without temporal and spatial limitations. As depicted in Figure 6, healthcare professionals can first input required information, and they can then predict the probability of there being severe, mild, and no adverse effects present when caring for at-risk patients, as shown in Figure 7.

## 4. Discussion

Fall severity can exert direct catastrophic percussion on patients and their families and indirect direct catastrophic percussion upon healthcare facilities and involved staff; thus, prevention of fall events should be dealt with due diligence. Therefore, prior knowledge of what constitutes the fall risk factors and what is the severity of falls are paramount issues for healthcare providers and facilities. In this study, we utilized machine learning techniques to predict the level of severity caused by patient falls. Knowing the risk factors of severity of patient falling events and also being able to predict the plausible severity of such fall events, healthcare facilities can improve patient safety. Likewise, they can better utilize limited resources to undertake proper interventions on the most needful patients. Among the seven algorithms adopted in our study, RF showed the best predictive performance over the remaining algorithms examined. Based on the RF algorithm, we built a web-based prediction support system which can unravel geographic and temporal constraints. Moreover, we also identify the top five fall severity risk factors, based accordingly on the SHAP value, including age, ability of independent activity, use of assistive devices, patient source, and fall history within the past 12 months aspect.

Several findings of this study are interesting and deserve further attention. First, prior patient safety studies that employed machine learning techniques largely relied on SVM [13, 23, 25, 27, 29]. The overall performance of SVM in our study is lower than that of RF. A plausible reason might be that prior studies included all forms of incident types, while our study focused only on the singularity of fall events. Further, previous studies also incorporated text mining techniques for incident reports while our study only included reportage of structured data.

Second, regarding the five important features identified in our study. Our study found that age is an important predictor of fall risk severity based on the SHAP value. This finding corroborates with prior evidence [2, 18, 24] which clearly demonstrated that fall rate frequently increased with patient age. A higher fall rate may indicate a greater chance of severe injury by fall occurrence. Further, patients with impaired mobility generally tend to be at high risk of falling when moving independently, potentially resulting in the occurrence of serious fall injuries. A prior survey reports that elderly patients without the ability of independent activity have 14 times more likelihood to report having 2 or more falls in the prior 12 months when compared with the elders without limitations on their mobility [43]. Several other investigations of fall risk factors have also shown mobility being of some importance [2, 17] and lend credence to our findings.

The use of assistive devices was identified as an important predictor for fall severity which is consistent with prior evidence [21]. Chen et al. [21] demonstrated that those patients who fell were more regular to use assistive devices than non-fallers. This pointed out that patients with walking aids were more likely to move independently and thus lowered the probability of severe fall risks.

Fall history has been found to be an important risk factor for predicting future falls [2, 17, 21]. Our study also confirmed that a fall history event within the past 12 months is an influential feature for predicting fall severity, which is consistent with the literature [2, 17, 21]. Special precautions should be provided for patients with a prior fall history.

This study also found that patient sources (i.e., inpatients, outpatients, or emergency department patients) play a key role in predicting the severity of falls. Prior evidence showed that those patients who fall were discharged after their index visit to emergency department. They had higher probability to revisit emergency department for a fall-related complaint when compared with non-fallers [44]. Other evidence [2–4] also reported several potential fall risk factors for inpatients. Based on our findings, it can thus be suggested that factors including age, ability to engage in meaningful independent activity, use of assistive devices, an incidence of fall history within the past 12 months, and patient source are important for the predictive determination of fall severity. All of these factors should be considered when healthcare facilities and providers are planning patient fall-prevention strategies.

Third, the fall severity prediction support system is web-based, easy-to-use, and user-friendly. This system can be assessed without time and space limitations and any device that can browse the Internet brings about accessibility. Further, this prediction system can be used as a clinical decision support tool for management of in-hospital fall patients served by frontline healthcare professionals. Once the probability of severity of fall events is identified, this information can be integrated into respective hospital information systems, and it can thus be used to inform the healthcare professionals how much effort they have to put in this post-occurrence of the accident. This would include, but is not limited to, the frequency of nurses' vital sign assessments and the requirement of further brain computer tomography, physical exams, etc.

Our data were extracted from a patient safety reporting system, based on the specification of Joint Commission of Taiwan [30], from one hospital in Taiwan. The main idea of reporting adverse incidents is anonymity, voluntariness, confidentiality, unaccountability, and mutual learning [30]. Such a practice is supportive towards encouraging healthcare professionals to proactively report any incidents in their sphere of activity. However, several study limitations must be mentioned. This practice of reporting may inhibit healthcare professionals from disclosing every incident since it is not mandatory, which may have potential impacts on the generalizability of our predictive model. Future research may collect incident data across hospitals or even countries to compare and contrast the findings of this study.

## 5. Conclusions

Patient falls have received much attention among healthcare facilities worldwide due to its plausible severe adverse effects to patients in aging populations. A fall event is one of the important, perhaps most preventable, incidents involving patient safety, and it should be handled cautiously. Based on this understanding, our study developed a fall severity prediction support system based on machine learning techniques. By comparing the performance of seven machine learning algorithms (MLR, NB, RF, SVM, XGBoost, DL, and Stacking), we chose an algorithm with the best predictive performance in terms of four metrics, including accuracy, F1-score, precision, and recall. Among the seven algorithms, RF outperformed the remaining algorithms in all four metrics. Moreover, we have also identified important features for predicting severity levels of falling, including age, ability of independent activity, use of assistive devices, a fall history within the past 12 months, and patient source. We then built a web-based severity prediction system by using RF algorithm and Flask package. By leveraging this predictive system, healthcare facilities can improve patient safety practices and better allocate limited resources to critical fall occurrences. Moreover, frontline healthcare professionals can use this prediction system while facing fall incidence and perform risk stratification that provides an adequate response to vulnerable patients. This will be beneficial to patients, healthcare professionals, family, and bedside caregivers alike.

## Figures and Tables

**Figure 1:** Study purpose.

**Figure 2:** Area under the receiver characteristic curve (AUROC) of random forest for the test dataset.

**Figure 3:** Confusion matrix of random forest for the test dataset.

**Figure 4:** Bar plot of mean absolute SHAP values.

**Figure 5:** Beeswarm plots.

**Figure 6:** Fall severity prediction support system.

**Figure 7:** Fall severity prediction results.

**Table 1:** A summary of patient safety studies applying machine learning techniques.

Source	Incident type	Purpose	Best learner	Performance	Data source
Ong et al. [23]	All	To automatically detect extreme-risk events in clinical incident reports	Support vector machine	AUC = 0.92, F-measures = 0.86, precision = 0.88, and recall = 0.83 for incident types	Clinical incident reports
Marschollek et al. [24]	Fall events	To derive comprehensible fall risk classification models	C4.5	Accuracy = 0.66, sensitivity = 0.55, specificity = 0.67, positive/negative predictive values = 0.15/0.94	Fall incident reports
Cheng and Zhao [25]	Medication	To predict drug-drug interaction	Support vector machine	AUROC = 0.67	DrugBank
Wang et al. [13]	All	To automate the identification of patient safety incidents in hospitals	Support vector machine	F-score = 0.78 for incident type and F-score = 0.87 for severity level	Incident reporting systems
Marella et al. [12]	All	To screen cases associated with the electronic health record	Naive Bayes	AUROC = 0.93, accuracy = 0.86, and F-score = 0.88	Patient safety reporting system and electronic health records
Fong et al. [26]	All	To identify health information technology-related events	Logistic regression	AUC = 0.93 and F1 score = 0.77	Patient safety event report
Comfort et al. [27]	Medication	To classify individual case safety reports within social digital media	Support vector machine	Accuracy = 0.78 and gKappa = 0.83	Individual case safety reports and social digital media
Liu et al. [28]	Fall events	To explore potential fall incident clusters	Clustering	N/A	Incident reporting systems
Evans et al. [29]	All	To determine the incident type and the severity of harm outcome	Support vector machine	AUROC = 0.89 for incident types and AUROC = 0.71 for severity of harm	Incident reporting systems
Wang et al. [14]	Fall events	To predict the severity of inpatient falls	Multi-view ensemble learning with missing values	AUC = 0.81	Incident reports
Wang et al. [15]	All	To identify incident types and severity levels	Convolutional neural network	F-scores >0.85	Incident reporting systems
Liu et al. [16]	All	To improve the classification of the fall incident severity level	Random forest	Macro-*F*1 = 0.73	Incident reporting systems

*Note.* AUC/AUROC denotes the area under the receiver operating characteristic curve and N/A denotes not available.

**Table 2:** Operational definition of variables.

Type of variable	Name	Measurement	Definition	Supported literature
Features	Gender	Discrete	(1): Male (2): Female	[1, 19]
	Age	Discrete	(1): 20–30 (2): 31–40 (3): 41–50 (4): 51–60 (5): 61–70 (6): 71–80 (7): ≥81	[1, 2, 18, 24]
	Patient sources	Discrete	(1): Inpatient (2): Outpatient (3): Emergency department	[4, 18]
	Fall history within the past 12 months	Discrete	(1): Yes (2): No	[2, 17, 19]
	Ability of independent activity	Discrete	(1): Independence (2): Partial independence (3): Full dependence	[2, 17]
	Companionship	Discrete	(1): Yes (2): No	[2, 21]
	Use of assistive devices	Discrete	(1): Yes (2): No	[21]

Target	Severity of falls	Discrete	(1): No adverse effect (2): Mild adverse effect (3): Severe adverse effect	

**Table 3:** Important model parameter setting.

Learner	Parameter	Best setting
Multinomial logistic regression	Solver	Newton-cg
	Penalty	l2
	C	2.2
	Tol	0.0001
Naïve Bayes	var_smoothing	0.123285
Random forest	max_features	6
	min_samples_leaf	2
	n_estimators	760
Support vector machine	Kernel	Rbf
	Gamma	2
	C	100
eXtreme gradient boosting	max_depth	9
	n_estimators	100
	colsample_bytree	0.9
	learning_rate	0.3
Deep learning	hidden_layer_sizes	(50, 100, 50)
	Activation	ReLu
	learning_rate	Adaptive
	Solver	Adam

**Table 4:** Patient characteristics.

Feature	Levels	2019		2020	
		Frequency	%	Frequency	%
Gender	Male	132	63.16	137	57.81
	Female	77	36.84	100	42.19
Age	20–30	10	4.78	8	3.38
	31–40	11	5.26	12	5.06
	41–50	15	7.18	26	10.97
	51–60	73	34.93	76	32.07
	61–70	59	28.23	58	24.47
	71–80	29	13.88	42	17.72
	≥81	12	5.74	15	6.33
Patient sources	Inpatient	167	79.90	202	85.23
	Outpatient	17	8.13	19	8.02
	Emergency department	25	11.96	16	6.75
Fall history within the past 12 months	Yes	153	73.21	176	74.26
	No	56	26.79	61	25.74
High risk of falling	Yes	194	92.82	217	91.56
	No	12	5.74	17	7.17
	Unevaluated	3	1.44	3	1.27
Ability of independent activity	Independence	72	34.45	85	35.86
	Partial dependence	128	61.24	141	59.49
	Full dependence	9	4.31	11	4.64
Companionship	Yes	51	24.40	66	27.85
	No	158	75.60	171	72.15
Use of assistive devices	Yes	111	53.11	129	54.43
	No	98	46.89	108	45.57
Severity of falls	Severe adverse effect	100	47.85	128	54.01
	Mild adverse effect	34	16.27	36	15.19
	No adverse effect	75	35.88	73	30.80

**Table 5:** Model performance assessments.

Dataset	Learner	Accuracy (SD)	F1 (SD)	Precision (SD)	Recall (SD)
Training	Multinomial logistic regression (MLR)	0.442 (0.028)	0.442 (0.028)	0.443 (0.029)	0.443 (0.028)
	Naïve Bayes (NB)	0.461 (0.026)	0.448 (0.026)	0.460 (0.028)	0.472 (0.024)
	Random forest (RF)	0.783 (0.008)	0.784 (0.007)	0.785 (0.007)	0.788 (0.008)
	Support vector machine (SVM)	0.771 (0.008)	0.771 (0.008)	0.774 (0.008)	0.776 (0.009)
	eXtreme gradient boosting (XGBoost)	0.778 (0.006)	0.779 (0.005)	0.781 (0.005)	0.784 (0.005)
	Deep learning (DL)	0.721 (0.016)	0.720 (0.017)	0.735 (0.013)	0.725 (0.019)
	Stacking (RF + SVM + XGBoost + DL)	0.756 (0.014)	0.754 (0.014)	0.760 (0.019)	0.763 (0.015)

Test	Multinomial logistic regression	0.426	0.397	0.402	0.416
	Naïve Bayes	0.426	0.426	0.444	0.500
	Random forest	0.844	0.850	0.839	0.875
	Support vector machine	0.823	0.828	0.817	0.851
	eXtreme gradient boosting	0.835	0.843	0.831	0.866
	Deep learning	0.751	0.743	0.725	0.773
	Stacking (RF + SVM + XGBoost + DL)	0.781	0.775	0.758	0.799

*Note.* SD denotes standard deviation.

## Data Availability

Data are not available due to ethical constraints.
